# Inhibition of SDF-1/CXCR4 Axis to Alleviate Abnormal Bone Formation and Angiogenesis Could Improve the Subchondral Bone Microenvironment in Osteoarthritis

**DOI:** 10.1155/2021/8852574

**Published:** 2021-05-28

**Authors:** Hanjun Qin, Xingqi Zhao, Yan Jun Hu, Shengnan Wang, Yunfei Ma, Siying He, Ke Shen, Haoyang Wan, Zhuang Cui, Bin Yu

**Affiliations:** ^1^Department of Orthopaedics, Nanfang Hospital, Southern Medical University, Guangzhou 510515, China; ^2^Guangdong Provincial Key Laboratory of Bone and Cartilage Regenerative Medicine, Nanfang Hospital, Southern Medical University, Guangzhou 510515, China

## Abstract

The pathogenesis of the osteoarthritis (OA) is complex. Abnormal subchondral bone metabolism is an important cause of this disease. Further understanding on the pathology of the subchondral bone in OA may provide a new therapy. This research is about to investigate the role of SDF-1 in the subchondral bone during the pathological process of OA. In vitro, Transwell was used to test the migratory ability of bone marrow mesenchymal stem cells (BMSCs) and human umbilical vein endothelial cells (HUVECs). Western blot presented the protein level after SDF-1 treatment in BMSCs and HUVESs. Alizarin red was used to assess the ability of osteogenic differentiation. To inhibit SDF-1 signaling pathway in vivo, AMD3100 (SDF-1 receptor blocker) was continuously delivered via miniosmotic pump for 4 weeks in mice after performing anterior cruciate ligament transaction surgery. Micro-CT, histology staining, immunofluorescence, immunohistochemistry, and TRAP staining were used to assess the role of SDF-1 on osteogenesis and angiogenesis in the subchondral bone. Our results showed that SDF-1 could recruit BMSCs, activate the p-ERK pathway, and enhance osteogenic differentiation. SDF-1 promoted the ability of proliferation, migration and tube formation of HUVECs by activating the ERK and AKT signaling pathways. In an animal study, inhibition of SDF-1/CXCR4 axis could significantly reduce subchondral osteogenesis differentiation and H-type vessel formation. Furthermore, the AMD3100-treated group showed less cartilage destruction and bone resorption. Our research shows that SDF-1 alters the microenvironment of the subchondral bone by promoting osteoid islet formation and abnormal H-type angiogenesis in the subchondral bone, resulting in articular cartilage degeneration.

## 1. Introduction

Osteoarthritis (OA) is the most common bone joint disease, characterized by the degeneration of cartilage which leads to pain and loss of function, affecting 9.6% of men and 18% of women over 60 years of age [1, 2]. The traditional treatment of OA includes pain management in the preliminary stage and arthroplasty in the end stage [3–5]. The effect of current pharmacologic therapies in altering the progression of OA is unsatisfactory. Arthroplasty surgery has its limitations including complications and even the possibility of adverse outcomes [2, 6]. Although aging, trauma, excessive mechanical load, and genetic factors have been reported to be associated with OA, the exact mechanisms remain unclear [7–9].

A functional unit in the joint consists of the articular cartilage and subchondral bone [10, 11]. The subchondral bone provides mechanical support, acting as a structural girder and shock absorber for the articular cartilage, and suffers bone remodeling constantly at the same time. The subchondral bone consists of the subchondral bone plate (SBP) and the subarticular spongiosa, separated by the cement line from the calcified zone of the articular cartilage [12, 13]. During OA development, aberrant MSC recruitment will interrupt coupled bone remodeling and form aberrant osteoid islets in the bone marrow [14]. Abnormal vascular congestion in the subchondral bone is reported as a pathological feature of OA. The aberrant osteochondral angiogenesis breaches the tidemark and aggravates OA progression [15, 16].The subchondral bone microarchitecture has been reported to change preceding the articular cartilage damage in OA [17–21]. All these imply that a change of the subchondral bone may be a trigger in OA progression. Aberrant osteoid islet and ostoechondral angiogenesis may play an important part in subchondral bone remodeling during OA.

Stromal cell-derived factor l (SDF-1) was found dramatically elevated in knee synovium from OA patients. In addition, compared with preoperative status, synovectomy significantly reduces the level of SDF-1, MMP-9, and MMP-13 in the serum [22]. SDF-l, also called CXCL12, is a chemokine in the CXC family, functioning by binding to its cell surface receptor, C-X-C chemokine receptor type 4 (CXCR4) [23, 24]. SDF-1 could activate CXCR4 and modulate various biological processes, such as cell proliferation, differentiation, chemotaxis, survival, and apoptosis [25]. Previous studies had reported CXCR4 promotes angiogenesis both in vitro and in vivo [26, 27]. Activation of the SDF-1/CXCR4 axis significantly promotes tissue regeneration, cardiomyocyte survival, and neovascularization after myocardial infarction and vascular disease [28]. Moreover, the SDF-1/CXCR4 axis plays an important role in the chemotaxis of stem cells and progenitor cells, as well as organ-specific homing [28, 29].

Although lots of researches studied on the relationship between SDF-1 and the cartilage [22, 30, 31], few literatures reported the role of SDF-1 in the subchondral bone during OA progression. Due to the subchondral bone microarchitecture destruction playing a crucial role in the early stage of OA, further study on the mechanism of the subchondral bone disordered remodeling is necessary. In current study, we attended to investigate the role of SDF-1 in the alteration of the microenvironment in the subchondral bone during the pathological process of osteoarthritis.

## 2. Materials and Methods

### 2.1. Cell Culture

The primary BMSCs were isolated from the femurs and tibias of four-week-old mice under sterile condition. The bone marrow cavity was flushed with MEM alpha medium; then, large tissues were removed with a 200-mesh nylon filter. The isolated bone marrow cells were cultured in MEM alpha medium which was supplemented with 10% fetal bovine serum (FBS), 100 U/ml penicillin, and 100 *μ*g/ml streptomycin. Primary human umbilical vein endothelial cells (HUVEC) were purchased from ScienCell (Carlsbad, CA) and cultured in DMEM with 10% FBS, 100 U/ml penicillin, and 100 *μ*g/ml streptomycin. All cells were cultured at 37°C in an environment with 5% CO_2_.

### 2.2. Western Blot

In the BMSC experiment, the control groups' BMSCs were cultured for 15 min in osteogenic inductive media. In the experimental groups, BMSCs were treated with 100 ng/ml SDF-1(Sigma, S5816) for 15 min with or without 2 hr pretreatment of 200 ng/ml AMD3100 (Abcam, ab120718) in osteogenic inductive media. In the HUVEC experiment, HUVECs were treated with 20 or 50 ng/ml SDF-1 for 30 min with or without 2 hr pretreatment of 200 ng/ml AMD3100.

After washing by phosphate buffer solution (PBS) for three times, protein from cells were extracted. An equal amount of proteins (30 *μ*g) was loaded onto 10% Tris/glycine gels for electrophoresis and transferred to a PVDF membrane. 5% nonfat milk was used to block for 1 hour at room temperature with shaking. Primary antibodies, anti-p-ERK (Affinity Bioscience, AF1015), anti-total Erk1/2 (Selleck, A5029), anti-p-Akt (HuaAn，ET1607-73), and anti-total AKT (A5023; Bimake), were, respectively, added to incubate at 4°C overnight. Then, TBST was used to wash the membrane for 3 times, each time for 10 minutes. Subsequently, the membrane was incubated with horseradish peroxidase-linked secondary antibodies. TBST was used to wash the membrane 3 times for 10 min each time again.

### 2.3. Transwell

The migration assay was designed using Transwell plates (Corning Costar, USA) with 6.5 mm in diameter and 8 *μ*m pore filters. In the controls, 1 × 10^5^ BMSCs or HUVECs in 200 *μ*l of DMEM containing 0.1% BSA were loaded in the upper chambers and the lower chambers treated with 500 *μ*l of DMEM containing 10% FBS. In the SDF group, the lower chambers were additionally treated with SDF-1 (100 ng/ml). In the AMD group, BMSCs in upper chambers underwent 2 hr pretreatment of 200 ng/ml AMD3100, and the lower chambers were also treated with SDF-1 (100 ng/ml). Following incubation for 15 h, cells in the upper chamber were removed and the membranes were fixed in 4% paraformaldehyde for 20 min. The cells that migrated to the lower side of the filter were stained with 0.1% crystal violet for 10 min and then observed under a light microscope.

### 2.4. Alizarin Red Staining

To assess osteogenic inductive ability of SDF-1, BMSCs were cultured in the osteogenic inductive medium and osteogenic differentiation was determined by Alizarin red staining. The SDF group was additionally added 100 ng/ml SDF-1 in osteogenic inductive media. In the AMD group, we pretreated BMSCs with 200 ng/ml AMD3100 2 hours and additionally added 100 ng/ml SDF-1 and 200 ng/ml AMD3100. After 28 days of osteogenic induced culture, mineral nodules were stained and evaluated by macroscopic and the microscopic observation.

### 2.5. Cell Proliferation and Cell Viability

The effects of SDF-1 on HUVEC proliferation and viability were assessed using the CCK-8 (Dojindo) assay. HUVECs were inoculated in 96-well cell culture plates (Costar, Cambridge, MA, USA) at the concentration of 5 × 10^3^ cells per well and maintained in DMEM (concluding 5% FBS) with SDF-1 (20 ng/ml, 50 ng/ml) or AMD3100 (200 ng/ml) for 1, 2, and 4 days. At each time point, HUVECs were treated with the CCK-8 reagent and incubated at 37°C for 2 h. Then, the absorbance in each well was measured at a wavelength of 450 nm using an automatic enzyme-linked immunosorbent assay reader (ELx800; BioTek Instruments Inc., Winooski, VT, USA). Proliferation was additionally assessed in a 5-ethynyl-2′-deoxyuridine (EdU) incorporation assay, by using the YF488 Click-iT EdU Imaging Kits (US Everbright Inc., C6015). SDF-1 at different concentrations (with or without AMD3100 200 ng/ml pretreatment for 2 hours) was administered by HUVECs for 4 days before addition of 10 *μ*M EdU for 2 h. Then, the click-iT reaction mixture was added, and nuclear redyeing was performed at last. OLYMPUS IX71 was used for photography and quantitative analysis.

### 2.6. Tube Formation

Each well of twenty-four-well plates were coated with 300 *μ*l Matrigel (BD, San Jose, CA) and incubated at 37°C for 20 min to solidify the Matrigel. After treatment with SDF-1 (20 ng/ml, 50 ng/ml) or AMD3100 (200 ng/ml) for 48 h, HUVECs were inoculated at the concentration of 1 × 10^5^ cells per well and incubated at 37°C for 12 h. Five randomly selected fields per well were photographed by Olympus IX71 digital camera. Tube formation was quantified by measuring the length of capillary structures using the software ImageJ.

### 2.7. Animals

Three-month-old male C57 Black6/J mice were obtained from the animal center of Southern Medical University. Mice were randomized into three groups: the ACLT group (*n* = 5) animals underwent anterior cruciate ligament transected (ACLT) on the left knee and were treated with PBS via constant infusion osmotic minipump; sham-operated group (*n* = 5) animals underwent sham surgery on the left knee; and AMD group (*n* = 5) animals underwent anterior cruciate ligament transected on the left knee and then treated with AMD3100 via constant infusion osmotic minipump for 4 weeks. The animal experiment was reviewed and approved by the Institutional Animal Care and Use Committee of the Southern Medical University, Guangzhou, China.

### 2.8. Surgery

To induce abnormal mechanical loading-associated osteoarthritis of the knee, the anterior cruciate ligament was transected using a surgical microscope and microsurgical technique as previously described [32]. The cartilage was protected from injury during the procedure. The left knee joints of the mice in the sham group were performed the same approach without the anterior cruciate ligament mutilation. All mice were allowed unrestricted activity, food, and water and housed under standard conditions in the Animal Facility of the Southern Medical University.

### 2.9. Delivery and Dose of AMD3100

A 1.2 cm transverse skin incision was made over the dorsal thorax. Blunt dissection was performed to create a subcutaneous pocket. The loaded Alzet osmotic minipump (model 1004, 0.11 *μ*l/hr Alza, Palo Alto, CA) was inserted in the subcutaneous pocket. Layer sutured and incision closed with 8-0 nylon after implantation. AMD3100 was filled the Alzet osmotic minipump and delivered at a rate of 180 *μ*g/day, which corresponds to steady serum level of 0.3 *μ*g/ml [33]. After 4 weeks of treatment, the animals were euthanized and the knee joints were collected.

### 2.10. Micro-CT

The knee joints of mice were dissected free of soft tissue, then fixed in 10% formalin overnight. The subchondral bone was scanned using high-resolution micro-CT (SkyScan 1172) and reconstructed the scanned images by image reconstruction software (NRecon v1.6). In the present study, sagittal views of the medial compartment of the tibial subchondral bone were used to perform the 3D histomorphometric analysis. The 3D structural parameters analysis of the tibial subchondral bone include bone mineral density (BMD), bone volume/total tissue volume (BV/TV), Tb.Th (trabecular thickness), Tb.N (trabecular number) Tb.Sp (trabecular separation), and structure model index (SMI).

### 2.11. Histopathological Examination

The knee specimen samples were harvested at 4 weeks postsurgery. Bone specimens were fixed in 4% buffered formalin for 48 hours. After the specimens were decalcified (10% EDTA for 21 days) and embedded in paraffin, sagittal sections were made from the medial side. The 4 *μ*m thick sections of the embedded specimens were stained by HE, immunofluorescence, immunohistochemistry, and TRAP staining. We use Olympus DP71 to perform histomorphometric measurements on the entire area of the tibial subchondral bone. There were 5 animals in each group. Three slides were randomly selected from each animal, and one full low-power field or three random high-power fields were selected for each slide for quantitative analysis of related indicators.

### 2.12. Immunochemical Examinations

For immunohistochemically staining, sections were incubated by primary antibody RUNX2 (Abcam, ab76956) overnight at 4°C after standard protocol. Horseradish peroxidase-streptavidin detection system was used to detect immunoreactivity and counterstaining with hematoxylin. Immunofluorescent staining was performed using a standard protocol, we incubated sections with primary antibodies: SDF-1 antibody (Santa Cruz, sc-74271), osterix (Santa Cruz, sc-393060), p-ERK (Affinity Bioscience, AF1015), CD31 (Abcam, ab222783), and Endomucin (Emcn, Santa Cruz, sc-65495) overnight at 4°C. A second antibody conjugated with fluorescence was added to the sample sections and incubated for 1 h at room temperature (RT).

### 2.13. Statistical Analysis

All in vitro experiments were repeated three times independently, and three random high-power fields were selected for quantitative analysis in each experiment. All data were presented as mean ± SD. Two-tailed unpaired Student's *t*-test was used for comparing two group parameters. One-way analysis of variance (ANOVA) was used for comparing multiple group parameters. Homogeneity of variance was tested first, and then, the differences between groups were assessed by post hoc multiple comparisons. Specifically, if no heterogeneity was observed, the Bonferroni test was used to assess the differences between groups. However, if heterogeneity did exist, the Welch test was used to test the equality of means and the Dunnett's T3 was used to assess the differences between groups. The investigators were blinded to allocation during experiments and outcome assessment. The level of significance was set at *P* < 0.05 and indicated by “^∗^” compared as denoted by bar, *P* < 0.01 was indicated by “^∗∗^” compared as denoted by bar. All data analysis was conducted with SPSS 22.0 analysis software (SPSS Inc.).

## 3. Results

### 3.1. Inhibition of SDF-1 Signaling Reduces Aberrant Subchondral Bone Formation and Attenuates Articular Cartilage Degeneration in Animal Experiments

To investigate the role of SDF-1 in the subchondral bone, we tested the level of SDF-1 in the subchondral bone in the ACLT group and sham operation group. Immunofluorescent staining showed that the level of SDF-1 elevated significantly in the subchondral bone of ACLT mice compared with sham controls (*P* < 0.01) (Figures 1(a) and 1(b)). Three-dimensional micro-CT images of the tibial subchondral bone from mice showed that there exists an abnormal bone formation in the ACLT group, while the abnormal bone formation feature in the subchondral bone was downregulated in the AMD group (Figure 1(c)). For micro-CT 3D analysis, BMD, BV/TV, Tb.N, and Tb.Th were significantly increased in the ACLT group compared with the sham operation control group. However, there is no difference between the AMD group and sham operation control group. We found that the mice treated with AMD3100 rescue these parameters to a normal level (Figures 1(d)–1(g)).

Safranin-O/fast green staining demonstrated that the ACLT group had more proteoglycan loss and articular cartilage degeneration than the AMD group (Figures 1(h) and 1(i)). H&E staining where calcified cartilage (CC) and hyaline cartilage (HC) thickness are marked by double-headed arrows showed that calcified cartilage in the ACLT group significantly increased, while the AMD3100 treatment group decreased the thickness of calcified cartilage (Figures 1(j) and 1(k)). These results indicated that the level of SDF-1 increased in OA. Inhibition of the SDF-1/CXCR4 axis effectively attenuated articular cartilage degeneration.

### 3.2. SDF-1 Recruits BMSCs and Promotes BMSC Osteogenic Differentiation In Vitro

Transwell was used to evaluate the migratory ability of BMSCs. Our result revealed that SDF-1 markedly induces the migration of BMSCs while migration was suppressed when pretreated with AMD3100 (*P* < 0.01) (Figures 2(a) and 2(b)). Western blot showed that the level of p-ERK1/2 was upregulated in the SDF-1 group. However, AMD3100-pretreated BMSCs showed significantly lower expression of p-ERK1/2, which suggests that SDF-1 activates the intracellular ERK phosphorylation in osteogenic differentiation of MSCs (Figures 2(e) and 2(f)). In addition, the Alizarin red staining showed that mineral nodules in the SDF-1 group significantly increased compared with the control group and AMD group (*P* < 0.01) (Figures 2(c) and 2(d)). From these results, we found that SDF-1 upregulates the level of p-ERK and promoted osteogenic differentiation in BMSCs. What is more, SDF-1 enhanced the ability of migration of BMSCs. All the results demonstrated a high level of SDF-1 promoted BMSC recruitment and osteogenic differentiation which led to more bone formation.

### 3.3. In Vivo, Inhibition of SDF-1 Signaling Reduces BMSC Recruitment and Osteogenic Differentiation and Bone Resorption

The immunofluorescent staining with nestin (a marker of adult BMSCs [34]) and osterix (a marker of osteoprogenitors) showed that a significant increase in the numbers of nestin-positive cells or osterix-positive osteoprogenitors in the subchondral bone marrow cavity in the ACLT group when compared with the AMD group (*P* < 0.01) (Figures 3(a)–3(d)). We confirmed p-ERK1/2 was upregulated in the ACLT group by immunofluorescent staining, and the level of p-ERK1/2 was decreased in the AMD group (Figures 3(e) and 3(f)). Additionally, immunohistochemical staining showed that the level of RUNX2 evidently increased in the subchondral bone in the ACLT group compared with the sham control group and AMD group (Figures 3(i) and 3(j)). The results of tartrate-resistant acid phosphatase (TRAP) staining revealed that the number of TRAP-positive osteoclasts in the subchondral bone was significantly increased in the ACLT group (*P* < 0.01) and decreased to normal when treated with AMD3100 (Figures 3(g) and 3(h)). These findings showed inhibition of the SDF-1/CXCR4 axis normalized the abnormal osteogenesis in the subchondral bone in OA.

### 3.4. SDF-1 Promotes HUVEC Migration and Proliferation and Upregulated the Level of p-ERK and p-AKT in HUVECs

The result of CCK8 showed that the inhibited SDF-1/CXCR4 axis attenuates the proliferation ability and cell viability of HUVECs (Figures 4(a) and 4(b)). In addition, the EdU experiment was consistent with the results of CCK8, and activation of the SDF-1/CXCR4 axis significantly promoted the proliferation of HUVECs (Figures 4(c) and 4(d)). In Transwell experiment, we found out that the migratory ability of HUVECs significantly increased after treated with SDF-1 (100 ng/ml) (Figures 4(e) and 4(f)). These results revealed that SDF-1 promoted HUVEC migration and proliferation.

### 3.5. In Vivo, Inhibition of SDF-1 Signaling Reduces BMSC Recruitment and Aberrant Blood Vessel Formation in Subchondral Bone

We analyzed the H-type vessels by performing double immunofluorescence staining for CD31 and endomucin [35]. We found that CD31-positive/Emcn-positive blood vessels were significantly increased in the subchondral bone in the ACLT group. Inhibition of SDF-1 signaling restored CD31-positive/Emcn-positive blood vessels similar to sham controls (Figures 5(a) and 5(b)). In addition, after treatment with SDF-1, HUVECs accelerated tube formation compared with the control. However, there are few tube formation after inhibiting the SDF-1/CXCR4 axis (Figures 5(c) and 5(d)). The western blot result showed SDF-1 activated the p-ERK and p-AKT signals (Figures 5(e) and 5(f)). Taken together, SDF-1 can effectively upregulate the levels of p-ERK and p-AKT in HUVECs and promote the vessel formation.

## 4. Discussion

Osteoarthritis is a common and disabling degenerative disease characterized by cartilage destruction and loss of joint function. Although degeneration of the cartilage is considered an important part in OA, recent studies believe subchondral bone deterioration exerts a central role in triggering a cascade of events which lead to cartilage degeneration, as well as the onset of OA [36]. Although subchondral sclerosis is considered an critical sign of OA, the integrity of the subchondral bone is important to maintain the function of the knee joint [37]. The subchondral bone provides mechanical support for the articular cartilage. Disordered bone remodeling in the subchondral bone plays an important part in OA progression.

SDF-1, also named pre-B cell-growth-stimulating factor (PBSF) or CXCL12, is a chemokine expressed by stromal cells and initially characterized as a growth-stimulating factor for a B-cell progenitor [38]. SDF-1 plays an important part in multiple processes during embryogenesis such as hematopoiesis, cardiogenesis, vascular formation, and neurogenesis [39]. In an adult, knockout of SDF-1 in mice leads to disruption of HSC homeostasis [40]. Previous studies demonstrated that SDF-1 was responsible for the homing and retention of hematopoietic stem cells in the bone marrow [41]. In OA, many studies believe that SDF-1 is mainly expressed by bone marrow stromal stem cells [42] and osteoblasts [43] in the bone but not produced by chondrocytes in the cartilage [22, 44]. Therefore, we believe that SDF-1 plays a crucial role in the regulation of the microenvironment of the subchondral bone. Our study showed that the abnormal increased of SDF was obviously closely related to the destruction of articular cartilage during the pathological process of osteoarthritis (Figures 1(a), 1(b), and 1(h)–1(k) ). Micro-CT analysis demonstrated that the subchondral bone of mice was in an anomalous remodeling status after ACLT operation. Inhibition of SDF-1 signaling was able to reduce aberrant subchondral bone formation. The 3D sagittal images presented that the subchondral bone was destructive in the ACLT-operated mice, while inhibited SDF-1 signaling could maintain the integrity of the subchondral bone (Figure 1(b)). In addition, blocking the SDF-1 signaling pathway could restore the BMD, BT/TV, Tb. Th, and Tb. N to normal (Figures 1(c)–1(f)).

In order to find out how SDF-1 specifically participates in the regulation of the subchondral microenvironment, we conducted in vitro experiments. After BMSCs treated with SDF-1 with or without AMD3100, Transwell test, Alizarin red experiment, and western blot were performed. Our results showed that SDF-1 could promote BMSC migration, and using AMD3100 to inhibit SDF-1/CXCR4 signaling significantly reduced the migration rate of BMSCs (Figures 2(a) and 2(b)). Alizarin red staining also confirmed that inhibition of SDF-1 signaling could significantly decrease BMSC osteogenic differentiation (Figure 2(c)). It is commonly agreed that the activated ERK pathway of MSCs could obviously promote osteogenic differentiation [45]. In addition, it has been reported that inhibition of the MAPK signaling pathway can effectively protect chondrocytes from damage caused by factors such as Sema4D, which indicate that the MAPK signaling pathway may play an important role in OA [46]. In the present study, we found out that SDF-1 could obviously activate the ERK signaling which may indicate that SDF-1 may have promoted BMSC migration and osteogenic differentiation through the ERK signal pathway. We considered during the OA pathology, one of the important reasons for the changes of the subchondral bone microenvironment is that the abnormal increase of SDF-1 leads to the increase of abnormal osteogenesis and the formation of osteophytes, thus changing the stress structure of the subchondral bone.

To further investigate the role of SDF-1 in changes of microenvironment in teh subchondral bone during OA, we observed the histomorphology of C57 mice in the control, ACLT, and AMD groups. The AMD groups inhibited SDF-1 signaling by constantly delivering AMD3100 via Alzet osmotic minipump after ACLT operation (AMD3100 was delivered at a rate of 180 *μ*A/day, which corresponds to steady serum level of 0.3 *μ*g/ml). In vivo, we found that the number of Nestin-positive cells and osterix-positive cells in the subchondral bone were reduced in the AMD group which means inhibition of SDF-1 signaling could effectively decrease the abnormal increase of BMSCs (marked by nestin^+^ cell) and osteoprogenitor cells (marked by osterix^+^ cell) in the subchondral bone (Figures 3(a)–3(d)). It is generally believed that the increase of BMSCs and bone progenitor cells will lead to increased osteogenic level in the subchondral bone. p-ERK and RUNX2 levels were significantly elevated in the ACLT groups but restored to normal after antagonizing the SDF-1 signaling pathway. Our study found that SDF-1 can significantly activate the ERK signaling pathway and induce abnormal bone formation in the subchondral bone in animal experiments, which is consistent with the results of cell experiments (Figures 3(e), 3(f), 3(i), and 3(j)). To maintain microenvironmental stability in the subchondral bone, a balance between osteogenesis and bone resorption is essential. Therefore, we tested TRAP-positive osteoclast activity in the subchondral bone and found that the inhibition of the SDF-1/CXCR4 signaling pathway significantly reduced the abnormal osteoclast activity in the subchondral bone. Overall, our animal experiments have demonstrated that an abnormal increase in SDF-1 is an important factor contributing to the imbalance of the subchondral bone microenvironment.

At present, abnormal angiogenesis in the subchondral bone leads to invasion of vasculature into the osteochondral junction is a hallmark of human osteoarthritis [46]. Type H vessels, characterized by high expression of endothelial markers CD31 and Emcn (CD31^hi^Emcn^hi^), produce a unique microenvironment to maintain perivascular bone progenitor cells and to link angiogenesis to bone progenitor cells [46]. Several previous studies suggested that neovessel formation in the subchondral bone is characterized by the development of osteogenesis-coupling type H vessels (CD31^hi^Emcn^hi^) [14, 47, 48]. In our experiment, we found that SDF-1 is closely associated with abnormal angiogenesis in the subchondral bone. SDF-1 significantly promoted the proliferation and activity of HUVECs (Figures 4(a)–4(d)). SDF-1 is also involved in the recruitment of HUVECs during the process of angiogenesis. Inhibition of the SDF-1/CXCR4 axis significantly suppressed HUVEC migration (Figure 4(e) and 4(f)). We believed that SDF-1/CXCR4 plays an important role in angiogenesis. Our experiment also confirmed this. In animal experiments, we found that H-type blood vessels marked by CD31^hi^Emcn^hi^ increased significantly in the ACLT group, while there was no statistically significant difference between the AMD3100 treatment group and the control group (Figures 5(a) and 5(b)). In vitro experiments, SDF-1 significantly accelerated the tubular formation ability of HUVECs and this phenomenon disappeared after antagonizing the SDF-1/CXCR4 signaling pathway (Figures 5(c) and 5(d)). Many studies have shown that activated the MAPK/ERK and PI3K/AKT signals can significantly promote angiogenesis in HUVECs [49, 50]. In our study, it was found that SDF-1 significantly upregulated the protein levels of p-ERK and p-AKT in HUVECs. Therefore, we considered that SDF-1 is likely to promote abnormal angiogenesis in the subchondral bone by mediating the MAPK/ERK and PI3K/AKT signaling pathways.

Our data suggest that SDF-1 alters the subchondral microenvironment by promoting abnormal osteogenesis (osteoid islet formation) and abnormal H-type angiogenesis in the pathologic progression of osteoarthritis. The osteoid islet formation in the subchondral bone alters stress distribution on the cartilago articularis, which leads to the degeneration of articular cartilage. In addition, angiogenesis promotes subchondral bone innervation, the neovessels and nerves begin to invade the avascular cartilage, leading to cartilage degeneration and painful symptoms [51]. Therefore, we believe that SDF-1 alters the microenvironment of the subchondral bone by promoting osteoid islet formation and abnormal H-type angiogenesis in the subchondral bone, resulting in articular cartilage degeneration.

Our current study also has drawbacks. For example, we did not further inhibit the MAPK/ERK or PI3K/AKT signaling pathway to verify the signaling mechanism of SDF-1 in the subchondral bone, and whether SDF-1 directly causes articular cartilage degeneration, etc. However, there are reasons to think that specific inhibition of SDF-1/CXCR4 in the early stage of osteoarthritis may improve and delay the pathological progression of osteoarthritis.

## Figures and Tables

**Figure 1:** (a, b) Immunofluorescent staining and quantitative analysis of SDF-1 in subchondral bone shows SDF-1 significantly elevates in the ACLT groups. Scale bar, 50 *μ*m. (c) Representative three-dimensional micro-CT images of sagittal views of the tibia subchondral bone medial compartment. (d–g) 3D parameter analysis of the tibia subchondral bone. (h, i) Safranin O and fast green staining shows proteoglycan loss and cartilage degeneration and the OARSI score for each group. Scale bar, 50 *μ*m. (j) H&E staining shows calcified cartilage (CC) and hyaline cartilage (HC) thickness marked by double-headed arrows. Scale bars, 50 *μ*m. (k) Quantitative analysis of CC and HC ratio in each group. ^∗^*P* < 0.05, ^∗∗^*P* < 0.01, and ^∗∗∗^*P* < 0.001.

**Figure 2:** (a, b) The microscopic observation of Transwell assay shows that SDF-1 significantly induces BMSC migration. Scale bar, 50 *μ*m. (c, d) The result of Alizarin red presents that SDF-1 promotes BMSC osteogenic differentiation. And inhibiting SDF-1 signaling by AMD3100 obviously reduces the number of mineral nodules. Scale bar, 100 *μ*m. (e, f) Inhibition of SDF-1 signaling downregulated p-ERK expression of BMSCs in the osteogenic inductive medium. S20 = SDF − 1 20 ng/ml, S50 = SDF − 1 50 ng/ml, *A* = AMD3100 200 ng/ml. ^∗∗^*P* < 0.01, ^∗∗∗^*P* < 0.001.

**Figure 3:** (a–d) Immunofluorescent staining and quantitative analysis of osterix+/nestin+ cells in the subchondral bone. Scale bar, 50 *μ*m. (e, f) Immunofluorescent staining shows p-ERK activity in the subchondral bone, inhibition of SDF-1 signaling downregulated p-ERK expression in vivo. Scale bar, 50 *μ*m. (g, h) Blocking the SDF-1 signaling reduces the number of TRAP+ osteoclasts in the subchondral bone. Scale bar, 100 *μ*m. (i, j) Immunohistochemical staining and quantitative analysis of RUNX2 in different groups. Scale bar, 100 *μ*m. ^∗∗^*P* < 0.01, ^∗∗∗^*P* < 0.001.

**Figure 4:** (a) The absorbance of CCK8 after treatment with SDF-1 (20 ng/ml, 50 ng/ml) or AMD3100 (200 ng/ml). (b) After treatment with SDF-1 (20 ng/ml, 50 ng/ml) or AMD3100 (200 ng/ml), the cell viability calculated by formula, cell viability (%) = [*A* (dosing) − *A* (blank)]/[*A* (0 dosing) − *A* (0 dosing)] × 100, *A* (dosing): absorbance of the well with cells, CCK8 solution and drug; *A* (blank): absorbance of the pore with medium and CCK8 solution, but no cells; *A* (0 dosing): absorbance of the well with cells, CCK8 solution, but no drug. (c, d) The proliferation effect of SDF-1 on HUVECs detected by EdU and quantitative analysis. Scale bar, 100 *μ*m. (e, f) The microscopic observation of Transwell assay shows that SDF-1 significantly induces HUVEC migration. S20 = SDF − 1 20 ng/ml, S50 = SDF − 1 50 ng/ml, *A* = AMD3100 200 ng/ml.^∗^*P* < 0.05, ^∗∗^*P* < 0.01.

**Figure 5:** (a, b) Double immunofluorescence staining shows inhibition of SDF-1 signaling restored CD31^+^Emcn^+^ blood vessels similar to sham controls. Scale bar, 100 *μ*m/50 *μ*m. (c, d) HUVECs treated with SDF-1(20 ng/ml, 50 ng/ml) or AMD3100 (200 ng/ml) in tube formation experiment. Scale bar, 50 *μ*m. (e) The result of western blot of HUVECs treated with SDF-1(20 ng/ml, 50 ng/ml) for 30 min with or without 2 hr pretreatment of AMD3100 (200 ng/ml). S20 = SDF − 1 20 ng/ml, S50 = SDF − 1 50 ng/ml, *A* = AMD3100 200 ng/ml. ^∗^*P* < 0.05, ^∗∗^*P* < 0.01, ^∗∗∗^*P* < 0.001.

## Data Availability

The datasets used to support the findings of this study are available from the corresponding author upon request.
